# Perilipin 2 Protects against Lipotoxicity-Induced Islet Fibrosis by Inducing Islet Stellate Cell Activation Phenotype Changes

**DOI:** 10.1155/2022/4581405

**Published:** 2022-07-06

**Authors:** Yunting Zhou, Yuming Wang, Chengming Ni, Huiying Wang, Junming Zhou, Bingying Wan, Huiqin Li, Fengfei Li, Rong Huang, Wei Xu, Ting Shan, Tingting Cai, Xiaoceng Kong, Bingli Liu, Xiaomei Liu, Zilin Sun, Jianhua Ma

**Affiliations:** ^1^Department of Endocrinology, Nanjing First Hospital, Nanjing Medical University, Nanjing, China; ^2^Department of Endocrinology, Zhongda Hospital, Institute of Diabetes, School of Medicine, Southeast University, Nanjing, China; ^3^Department of Cadre Gastroenterology, Jinling Hospital, Medical School of Nanjing University, Nanjing, China; ^4^Department of Nephrology, Changzhou Hospital of Traditional Chinese Medicine Affiliated to Nanjing University of Chinese Medicine, Changzhou, China; ^5^Department of Endocrinology, Xuzhou Central Hospital, Xuzhou Institute of Medical Sciences, Xuzhou Clinical School of Nanjing Medical University, Xuzhou, China

## Abstract

**Aims:**

We explored whether and how perilipin 2 (*Plin2*) protected islets against lipotoxicity-induced islet dysfunction by regulating islet stellate cells (ISCs) activation.

**Methods:**

Six-week-old male rats were given a high-fat diet or a control diet for 28 weeks. Glucose metabolic phenotypes were assessed using glucose/insulin tolerance tests, masson, and immunohistochemical staining. ISCs activation levels were assessed from rats and palmitic acid- (PA-) treated cultured ISCs by immunofluorescence, Oil red O staining, electron microscopy, quantitative PCR, and western blotting. Changes in ISCs phenotype of activation degree and its underlying mechanisms were assessed by target gene lentiviral infection, high-performance liquid chromatography (HPLC), and western blotting.

**Results:**

Obese rats showed glucose intolerance, decreased endocrine hormone profiles, and elevated expression of *α*-smooth muscle actin (*α*-SMA), a polygonal appearance without cytoplasmic lipid droplets of ISCs in rats and isolated islets. PA-treated cultured ISCs exhibited faster proliferation and migration abilities with the induction of mRNA levels of lipid metabolism proteins, especially *Plin2*. The overexpression of *Plin2* resulted in ISCs “re-quiescent” phenotypes associated with inhibition of the Smad3-TGF-*β* signaling pathways.

**Conclusions:**

Our observations suggest a protective role of *Plin2* in weakening ISCs activation. It may serve as a novel therapeutic target for preventing islet fibrosis for T2DM.

## 1. Introduction

Type 2 diabetes mellitus (T2DM) is a prevalent chronic metabolic disease associated with progressive islet dysfunction [1]. Ectopic fat deposition and excessive lipid droplets (LDs) in the cytoplasm of cells promote impaired glucose-stimulated insulin secretion, reduce insulin storage, inhibit pro-insulin synthesis, increase pancreatic fibrosis, and accelerate islet cell apoptosis [2–4]. Our previous studies showed that stellate cells in islets, named islet stellate cells (ISCs), which are rich in LDs and positive for desmin and GFAP expression under physiological conditions, proliferate fast and generate the fibrotic extracellular matrix (ECM) when activated by various pathological stimuli. Furthermore, ISCs show specific expression of *α*-smooth muscle actin (*α*-SMA), and secretion of collagen I (Col I), fibronectin (FN), and other ECM components that induce the formation of islet fibrosis with a parallel disappearance of LDs, consequently leading to T2DM [5, 6]. However, the underlying pathogenesis and mechanism of ISCs activation have not yet been investigated.

In cells from mammalian, LDs were regarded as a fuel supplier for energy support and as a lipolytic barrier for avoiding cellular lipotoxicity via the regulation of LD lipolysis [7]. Therefore, LDs, along with LD-associated proteins, are responsible for maintaining lipid metabolism homeostasis [8]. The perilipin family is a group of key LD-associated proteins, including enzymes for fat synthesis and decomposition, LD transporters, and fusion-related molecules involved in signal transduction. Among them, five members have been identified, namely, perilipin 1 (*Plin1*) to perilipin 5 (*Plin5*) [9]. This family of proteins is a marker molecule on the surface of LDs in eukaryotic cells and plays a critical role in regulating LD metabolism and maintaining intracellular lipid balance [10, 11]. The liver mainly expresses perilipin 2 (*Plin2*), perilipin 3 (*Plin3*), and *Plin5*, among which *Plin2* is highly expressed [12]. Some studies found mice on a high-fat diet (HFD) showed decreased liver TG and increased hepatic insulin sensitivity after *Plin2* antisense oligonucleotide treatment or after liver-specific *Plin2* knockout [13, 14]. In the pancreas, the majority of islet neutral lipid staining was shown to co-localize with PLIN2 and PLIN3 in human adult normal and T2DM patients [15]. Recently, Roland Stein et al. found [16] glucose-stimulated insulin secretion was blunted in *Plin2* knockdown EndoC-*β*H1 cells and improved in *Plin2* overexpression cells, suggesting LD accumulation regulated by perilipin levels is a critical signaling molecule to impact islet cell activity. However, the role of perilipin family in regulation of the ISC phenotype is unclear.

Our present study aimed to define the specific mechanism underlying the association between the perilipin family and ISCs phenotype, especially concerning the suppression of ISCs activation. Our findings will provide new insights into the underlying molecular mechanism of ISCs activation pathological process and novel target therapy for preventing its adverse effects on islets.

## 2. Materials and Methods

### 2.1. Animals

Sprague-Dawley rats (male, 6-week-old) were purchased and housed under standard conditions at constant temperature with a half-half light/dark cycle. All animals were randomly assigned to an obese group fed a HFD (*n* =12, 60% fat/total kcal) and a control group fed a commercial rodent chow diet (*n* =12, 10% fat/total kcal) for 28 weeks. Random blood glucose levels and body weight were detected weekly. All animal studies were established by the Research Animal Care Committee of Nanjing Medical University. All procedures of animal experiment were performed according to the Guide for the Care and Use of Laboratory Animals (NIH No. 8023, revised 1978).

### 2.2. ISC Isolation and Expansion

Islets from obese and control rats were obtained by digestion using collagen P solution (1 mg/mL; Sigma, USA) with following on purification on LSM density gradients (MP, CA, USA), and subsequently handpicked with 20 *μ*L pipettes [17]. ISCs were grown after islet attachment and cultured in Dulbecco's modified Eagle's medium/F12 supplemented with fetal bovine serum and penicillin-streptomycin (Gibco, Grand Island, NY, USA) using the standard protocol described in our previous article [18]. Cells prepared at 3-6 passages were used for further experiments.

### 2.3. Intraperitoneal Glucose Tolerance Test (IPGTT) and IP-Insulin Tolerance Test (IPITT)

For the IPGTT experiment, after fasting for 12 h before the experiment, blood samples from the tail vein of mice were harvested and measured at 0, 15, 30, 60, and 120 min followed by administering D-glucose (2 g.kg-1) using a glucose monitor (Bayer, Geneva, Switzerland). For the IPITT experiment, the rats fasted for 4 h before the experiment, and blood samples were obtained at the same points after insulin administration (1 IU.kg-1). Areas under the curve (AUC) of the blood glucose-time point function were obtained and calculated by Sigma Plot software (Systat Software, CA, USA). The value of homeostasis model assessment insulin resistance (HOMA-IR) was assessed through previously published procedures [17].

### 2.4. Western Blotting

ISCs were divided into treated and control groups, with PA-mixed medium (300 *μ*M) or with 0.05% BSA for 48, 72, and 96 h, respectively. At different in vitro culturing times, experiments were performed using the standard protocol [19] with the primary antibodies specific for the following proteins: rabbit anti-PLIN2 (Cat#ab108323, Abcam, UK), rabbit anti-PLIN3 (Cat#ab47638, Abcam, UK), Col I (Cat#ab34710, Abcam, UK), rabbit anti-FN (Cat#ab2413, Abcam, UK), rabbit anti-perilipin 4 (PLIN4) (Cat#10694-1-AP, Proteintech, USA), mouse anti-PLIN5 (Cat#sc-514296, Santa Cruz, USA), mouse anti-*β*-actin (Cat#TA811000, Origene, China), mouse anti-*α*-SMA (Cat#A2547, 1 : 3000, Sigma, USA), rabbit anti-P-Smad3 (Cat#9520, CST, USA), rabbit anti-Smad3 (Cat# 8685S, CST, USA), and rabbit anti-TGF-*β* (Cat#3711, CST, USA). Horseradish peroxidase- (HRP-) conjugated goat anti-rabbit (Cat#SE134, Solarbio, China) or anti-mouse (Cat#SE131, Solarbio, China) antibody was used as the secondary antibody. Quantitative analysis of proteins was performed using enhanced chemiluminescence (Millipore, USA) and Image J software (National Institutes of Health, MD, USA), respectively.

### 2.5. Immunohistochemistry and Immunofluorescence

Consecutive tissue sections were fixed in 4% paraformaldehyde with paraffin embedded. After blocked with 5% bovine serum albumin, the sections were incubated with a rabbit anti-insulin (Cat#ab181547, Abcam, UK)/glucagon (Cat#ab92517, Abcam, UK)/*α*-SMA antibody (1 : 200) at 4°C overnight. Following the washing step, sections were incubated with HRP-conjugated anti-rabbit antibody at room temperature for 1 h; immunohistochemistry was performed with DAB and counterstained with hematoxylin. Goat anti-mouse IgG H&L (Alexa Fluor® 594) (Cat#ab150116, Abcam, UK) antibodies (1 : 3000) were used as the secondary antibody. Immunofluorescence was performed as described previously [17] to evaluate *α*-SMA expression in islets. Masson trichrome staining was performed according to standard protocols [20].

### 2.6. Cell Viability, Migration, and Proliferation Assays

For the wound healing experiment, 3 × 10^5^ ISCs in each 6-well plate were grown to 70%-80% confluence, then the monolayers of cells were scraped off using 20 *μ*L pipette tip. After 24 h incubation, the cells that migrate into boundaries of the wound were manually counted. The area of ISCs migration was visualized and calculated under light microscopy using Image J software. For the CCK-8 experiment, cells were suspended at a final concentration of 2 × 10^3^/well and incubated for 24, 48, and 72 h, respectively. Thereafter, 10 *μ*L CCK-8 reagent (Keygen, Biotech) was added to 100 *μ*L standard serum-free medium. After incubating for 1 h at 37°C temperature, the absorbance of each well was measured using auto microplate reader (BioTek, Inc., USA).

### 2.7. Electron Microscopy (EM)

Freshly differentiated ISCs were fixed with control medium or induced medium in 2.5% glutaraldehyde containing 2.0% paraformaldehyde in phosphate buffer (adjusted pH to 7.4) for 1 h at 4°C. After rinsing in phosphate buffer, the cells were postfixed in 1% cacodylate-buffered osmium tetroxide at room temperature for 2 h and then dehydrated in a graded ethanol series (30%, 50%, 70%, 95%, and 100%). Following transferred to propylene oxide, the cells were embedded in epon. Ultrathin sections at 60-80 nm thick were placed on 200 mesh copper grids coated with formvar-carbon and stained with uranyl acetate and lead citrate. Microphotographs were obtained and analyzed using H-600-4 system (Hitachi, Japan).

### 2.8. qPCR Quantification

Total RNA from cells was obtained and isolated using TRIzol reagent (Life Technologies, USA), and each tube of RNA (1 *μ*g) was reverse transcribed with HiScript RT SuperMix kits (Vazyme, China). Then, the DNA was used to perform qPCR assay using SYBR Green PCR master mix kits (Vazyme, China). Specific mRNA primers of rat (Table 1) were designed at the GenBank database. PCR was performed with the following conditions: 95°C for 30 s, then 40 cycles of 95°C for 10 s and 60°C for 30 s using the Step One Real-Time PCR System (Applied Biosystems, Foster City, CA, USA). Relative mRNA expression was quantified using the *ΔΔ*Ct method.

### 2.9. Gene Transfection

Lentiviral vectors of target gene-*Plin2* overexpression were constructed by GenePharma company (Shanghai, China). ISCs from passage 6 were infected with *Plin2* overexpression vector at the best multiplicity of infection as the experiment group, and these transfected with empty vector were treated as control groups. Means of an inverted fluorescence were observed under the fluorescent microscope. Stable cell clones were selected by mixed medium supplemented with 2 *μ*g/mL puromycin for 6 days. The transfection efficiency of cells was estimated with qPCR and western blot analyses.

### 2.10. Lipid Accumulation Observation

Cell retinol levels were measured using a previously described method [17]. Triglyceride (TG) content was measured using commercial TG kits (Jiancheng Technology Co., China) following the manufacturer's instructions. All levels of retinol and TG were normalized to the protein concentration in the cells. Oil red O staining was conducted by incubating 4% paraformaldehyde-fixed material for 30 min at room temperature with Oil red O solution in isopropanol (Sigma, USA). The Oil red O positive staining area in images of cells in each well culture plate was converted Image J in our previously described method [19].

### 2.11. Statistical Analysis

Data are expressed as the mean ± S.E at least three independent experiments. Differences were evaluated and reported using Student's *t*-test and one-way ANOVA test post hoc analysis, respectively. Statistical significance was calculated at *P* < 0.05. All statistical analyses were determined using GraphPad Prism 6.0 statistical software (GraphPad Software, San Diego, CA).

## 3. Results

### 3.1. Effect of HFD on Islet Morphology and Function

Twenty-eight weeks of HFD feeding significantly aggravated body weight and serum insulin concentration (Figure 1(a)). We also detected glucose intolerance in obese rats, showing that blood glucose levels 15-120 min after glucose challenge were elevated. Although the random blood glucose levels in rats with or without HFD feeding were not influenced, modest but significant glucose intolerance with elevated HOMA-IR was shown in HFD-fed rats (Figures 1(b) and (d)). As shown in Figure 1(c), pancreatic islets in control diet-fed rats were mostly round with smooth contours. In contrast, islets in HFD-free rats showed abnormal disorder of cells with noncircular borders, and the number of glucagon- and insulin-positive cells was markedly decreased than those in the control rats. Masson's stained tissue histological analysis revealed an abnormal collagen arrangement in obese rats compared to the uniform deposition observed in control rats. Insulin immunoreactivity of the islets from obese rats also decreased while it was accompanied by upregulation of *α*-SMA in double immunofluorescence labeling, indicating ISCs activation (Figure 1(e)). Ultrastructural studies have shown that ISCs in control rats exhibit characteristics compatible with quiescent ISCs, namely, few LDs and abundant fibers in the extracellular compartment. The ISCs in obese rats displayed characteristics compatible with activated ISCs, namely, concomitant disappearance of the LDs and extensive collagen fibers in the extracellular compartment (Figure 1(f)).

### 3.2. Effect of High-Fat Diet on ISCs Bio-Phenotype *In Vivo*

As shown in Figure 2(a), the rate of ISCs outgrowth was markedly faster in HFD-fed rat islets cultured in medium than in those from control rats. One of the major changes of phenotypic characteristics of ISCs activation is the loss of LDs in cytoplasm. Following their activation status, ISCs isolated from HFD-fed rats also showed lower LDs content per cell than those isolated from controls at different time points (Figure 2(b)). Immunofluorescence showed more abundant *α*-SMA protein expression in ISCs from HFD rats than in ISCs from controls (Figure 2(c)).

### 3.3. Effect of PA on ISCs Bio-Phenotype *In Vitro*

After 48 h of incubating ISCs with PA (300 *μ*M), the upregulation protein expression of *α*-SMA, FN, and Col I was detected by western blotting, and this phenomenon continued until 96 h (Figure 3(a)). Furthermore, we also performed the wound healing migration assay to compare the migration rates of PA-treated ISCs and control ISCs. The results showed that PA-treated ISCs cultured in medium had a significantly faster migration rate than that of the control ISCs (Figure 3(b)). Similarly, PA-treated ISCs had significantly higher viability rates than control ISCs (Figure 3(c)).

### 3.4. Effect of PA on LDs-Associated Protein Expression in ISCs

After ISCs were treated with 300 *μ*M PA, the mRNA levels of lipid metabolism markers, such as peroxisome proliferator-activated receptor *γ* (*Pparγ*) and its target regulators-acyl-coenzyme A dehydrogenase 8 (*Acad8*), carnitine acyltransferase 1*α* (*Cpt1α*), acyl-coA thioesterase 1 (*Acot1*), and perilipin family members (*Plin2*, *Plin3*, *Plin4*, *Plin5*), decreased in a time-dependent manner relative to the control group, with *Plin2* being the least expressed (Figure 4(a)). The western bolt results showed that PA treatment in cultured ISCs induced protein levels of PLIN2 and Plin4 increased rather than PLIN3 and PLIN5 (Figure 4(b)).

### 3.5. Effect of *Plin2* Overexpression Weakening ISCs Activation via Smad3-TGF-*β* Signaling Pathway

We overexpressed *Plin2* in ISCs via lentiviral transduction to explore the effect of *Plin2* on ISCs phenotype. The results of changes of morphology and LDs content in these cells showed that ISCs overexpressed *Plin2* gene had a classical polygonal appearance similar to that of quiescent ISCs and expressed increase of protein of PLIN2 and reduction of protein of FN, Col I, and *α*-SMA compared with negative control (NC) ISCs (Figures 5(a) and (b)). We further investigated that lipid accumulation of triglyceride (TG) rather than retinyl ester was significantly increased in ISCs overexpressing *Plin2* than those in NC ISCs both in Figure 5(c). The abundance of fibrogenesis in ISCs overexpressing *Plin2* prompted us to assess the activation state of the classic fibrogenesis signaling pathways-Smad3-TGF-*β*. We found a 1.8-fold reduction in the Smad3 signaling pathway in ISCs overexpressing *Plin2* compared with NC ISCs. Similarly, TGF-*β* levels were decreased by 43% in overexpressed ISCs (Figure 5(d)). Thus, the results showed that *Plin2* inhibits ISCs activation through the Smad3-TGF-*β* pathways.

## 4. Discussion

The aim of this present study is to investigate the effects of perilipin family on lipotoxicity-induced islet dysfunction by mediating ISCs activation and its intracellular signaling mechanism. Our data showed that high fat and PA treatment increased the outgrowth rate of ISCs both *in vivo*, and induced accelerated cell migration and cell viability, elevated expression of *α*-SMA, and increased secretion of extracellular components *in vitro*. Furthermore, the above effects were associated with elevated levels of functional perilipin family active metabolites, especially *Plin2*, with the inactivation of Smad3 signaling pathway. To our knowledge, this is the first report to reveal the effects of the perilipin family on ISCs activation induced by lipotoxicity.

Increasing evidence points toward a strong association between the distribution of excess fat in obese patients with T2DM [21–23]. In the present study, we found that rats fed the HFD exhibited decreased insulin sensitivity, increased HOMA-IR values, and larger AUC of IPGTT and IPITT relative to those in controls rats. Furthermore, we used double immunofluorescence and electron microscopy to determine whether HFD induces phenotypic changes in ISCs in islets. The biological appearance from classical polygonal to fibroblast-like and upregulation of *α*-SMA immunoreactivity of the islets indicate ISCs activation. Emerging evidence showed that ISCs activation is the key issues for islet fibrosis under pathological conditions [6, 18, 24]. Our study also showed that ISCs grown from obese rat islets lost their cytoplasmic LDs more rapidly than those grown from normal rat islets. The elevated rate of ISCs outgrowth from the islets, viability of ISCs, migration rate of ISCs, and *α*-SMA expression of ISCs suggested the activation of obese rat ISCs, all of which are contributed to the fibrotic transformation process [25]. These results indicate that dietary high-fat supplementation for 28 weeks induced a positive relationship between *α*-SMA expression and ISCs in obese rats. These observations are consistent with previous studies that showed in diabetic environment, the activation of ISCs leads to increase in ISC-derived secretory products and influences islet function [5, 6, 19, 26]. Our group previously found that ISCs were similar but not identical to pancreatic stellate cells (PSCs) [27]. Given the developmental biological and anatomical location of ISCs, we believe that ISCs may contribute significantly to islet fibrosis. Thus, understanding the underlying molecular mechanism resulting in the quiescent state of ISCs may prevent its adverse effects on islet function.

To extend these observations, we explored the important role of LD-associated protein molecules in maintaining the quiescent phenotype of ISCs. Adipogenesis is known as an organized multistep process that requires the sequential activation of many transcription factors, including *Pparγ*, which are essential for maintaining stellate cells in their quiescent state [28–30]. *Pparγ* is considered a central regulator of lipid metabolism to maintain the adipocyte phenotype by directly binding to and transactivating response elements in several adipocyte-specific genes [31]. Recently, novel modes of LDs growth (including rapid/homotypic as well as slow/atypical LD fusion) have been revealed and essential proteins (e.g., the perilipin family) have been identified [32, 33]. Meanwhile, LDs mature by inhibiting neutral lipid core formation and decreasing *Plin2* and *Plin5* expressions via downregulation of *Pparγ* [34]. Under palmitate overload, upregulation of *Plin5* promotes LDs storage and alleviates lipotoxicity in INS-1 *β*-cells with improved cell apoptosis and *β*-cells function [35]. While exploring the role of the perilipin family in regulating the ISCs phenotype, we first found *Pparγ* and perilipin proteins, especially PLIN2, to be associated with decreased functional LDs active metabolites levels, which serve as key molecular events for lipotoxicity-driven ISCs activation. Recently, the protective effect of *Plin2* in human *β* cells against lipotoxic-induced cellular autophagic flux and reduces endoplasmic reticulum stress has been reported [15, 16, 36]. *Plin2* overexpression restored the polygonal appearance of quiescent ISCs with LDs re-formation and reduced the activation degree and ECM synthesis, producing a resting-state phenotype. This result is consistent with previously published reports showing that ligand-activated *Pparγ* upregulates *Plin2* gene expression and activity of the *Plin2* promoter to regulate the function of *Pparγ* on lipid storage at the cellular level [37]. Hence, our observations firstly showed that LD-associated protein molecules are essential for maintaining a quiescent ISCs population, suggesting that cell-based strategies that block ISCs activation potential could effectively remodel the ISCs bio-phenotype.

Additionally, our study provides insights into the intracellular signaling mechanisms underlying *Plin2*-mediated inhibition of ISCs activation. The results demonstrated that phosphorylation and activation of Smad3 reduced with *Plin2* overexpression in ISCs. Identifying these signaling pathways as targets for *Plin2* in ISCs is in agreement with our previous study and other reports, showing that the Smad-TGF-*β* pathway could be activated in ISCs from patients with diabetes [5]. Therefore, Smad3 signaling, one of the key pancreatic fibrosis parameters, is also a switch molecule of ISCs activation, as well as PSCs [5, 38]. Although these findings support that *Plin2* is crucial for inhibiting ISCs activation in the HFD-lipotoxic environment, the specific mechanism underlying needs further exploration. It is also required to investigate the effect of *Plin2* in association with ISCs activation using transgenic models to elucidate this process in diabetes pathogenesis; future studies should also determine whether accumulation in ISCs affects lipid homeostasis in islets and the insulin-resistant state in other tissues; what's more important is when and how the link and signals crosstalk are changed between ISCs and islet cells may answer how changes of LDs levels in ISCs regulate islet cell frangibility to lipotoxicity.

In summary, this study identified that this population of ISCs is activated toward to fibrotic phenotype by exposure to a lipotoxic environment. ISCs activation could be inhibited by *Plin2*, which participate in the regulation of the specific mechanisms with Smad3 signaling pathways to prevent ISCs activation fibrotic phenotype. These findings help us to clarify new targets for preventing or treating diabetes.

## Figures and Tables

**Figure 1:** Lipotoxicity induces glucose metabolic phenotypes damage and ISCs activation in vivo. (a) Body weight and circulating insulin content were detected from HFD and control rats. (b) Islet function of HFD and control rats was analyzed via IPGTT/IPITT experiment and HOME-IR value calculation. (c) Representative images of insulin/glucagon and masson's trichrome stained in pancreatic islets from HFD and control rats. (e–f) Representative images of insulin and *α*-SMA double-stained and electron microscopy in pancreatic islet sections from HFD and control rats. Quantification of *α*-SMA fluorescent signals was measured using Image Pro Plus software. Magnification: 40x, 10000x, 20000x; scale bars: 50 *μ*m, 1 *μ*m, 0.5 *μ*m. ∗*P* < 0.05, ∗∗∗*P* < 0.001. Error bars shown as ± SE of *n* =12 mice per group.

**Figure 2:** The phenotype changes of ISCs from HFD rats at different in vitro culturing time. (a) Relative light microscopy micrographs of ISCs outgrowth rates from HFD and control rats at different culture time point (0 h, 48 h, 96 h, and 120 h). (b) Relative Oil red O staining of lipid droplets images of ISCs from HFD and control rats at different in vitro culturing time (48 h and 96 h). (c) Immunofluorescent staining of *α*-SMA protein expression in ISCs from HFD and control rats. Magnification: 40x; scale bars: 50 *μ*m. ∗∗∗*P* < 0.001, ∗∗∗∗*P* < 0.0001. Error bars shown as ± SE of *n* =12 mice per group.

**Figure 3:** Lipotoxicity promotes the activation of ISCs in vitro. (a) The protein expression of *α*-SMA, Col I, and FN in ISCs with PA treatment for 48 h, 72 h, and 96 h. (b) The wound healing migration assay was measured in cultured ISCs from HFD and control rats for the migration rate. (c) The proliferation rat assay was measured using CCK8 in cultured ISCs from HFD and control rats. ∗*P* < 0.05, ∗∗*P* < 0.01. Error bars shown as ± SE of three independent repeated experiments.

**Figure 4:** PA decreases LDs-associated protein expression of ISCs. (a) The mRNA expression of LDs metabolism markers and its related proteins (*Plin2*, *Plin3*, *Plin4*, *Plin5*, *Pparγ*, *Acda8*, *Cpt1α*, *Acot1*) expression in ISCs were analyzed by q-PCR with PA treatment for 24 h, 48 h, and 72 h. (b) The protein expression of perilipin family and its (PLIN2, PLIN3, PLIN4, PLIN5) was detected by western blotting. ∗∗∗*P* < 0.001, ∗∗∗∗*P* < 0.0001. Error bars shown as ± SE of three independent repeated experiments.

**Figure 5:** *Plin2* overexpression reverses ISCs phenotype via proliferation and fibrogenesis signaling pathways. (a) Representative photomicrographs of phenotype change in activated ISCs transduced with *Plin2* gene overexpressed or NC. (b) The protein expression of *α*-SMA, Col I, and FN in ISCs overexpressed *Plin2* was detected by western blotting. (c) The lipid accumulation observation was measured in ISCs overexpressed *Plin2*. (d) The protein expression of Smad3-TGF-*β* in ISCs overexpressed *Plin2* was detected by western blotting. Magnification: 40x; scale bars: 50 *μ*m. ∗∗*P* < 0.01, ∗∗∗*P* < 0.001, ∗∗∗∗*P* < 0.0001. Error bars shown as ± SE of three independent repeated experiments.

**Table 1:** Sequences of rat specific primers used for qPCR.

Gene	Primer sequence (5′-3′)	
*Plin2*	F: ATTCTGGACCGTGCCGATTT	R: ATCCTTTGCCCCAGTTACGG
*Plin3*	F: TCATCAACAGTGTCTGGGGC	R: CTGAACACACTGAGTGCCTG
*Plin4*	F: CCCTTGTCCATCAGCTCCAC	R: CAAGTGGAGGGTTTTGCTGC
*Plin5*	F: GCTCTGCACTCAGGGATCTG	R: CACGCCTGTGACACTTTTGG
*Pparγ*	F: AGCATGGTGCCTTCGCTGATGC	R: AAGTTGGTGGGCCAGAATGGCA
*Acda8*	F: TGTGGATGTGATGCGGAAGG	R: TCAGTCCCAATCCTGTTGGC
*Cpt1α*	F:GGTCAACAGCAACTACTACG	R:TGAACATCCTCTCCATCTGG
*Acot1*	F: GACCACAACTGGAAGAGCGA	R: ACTTTTCCTGCCAAAACCATCA
*β-actin*	F: CCCTGAAGTACCCCATTG	R: TACGACCAGAGGCATACAG

## Data Availability

All data has been included in this article.
